# Leashes, Litterboxes, and Lifelines: Exploring Volunteer-Based Pet Care Assistance Programs for Older Adults

**DOI:** 10.3389/fpsyg.2022.873372

**Published:** 2022-04-26

**Authors:** Kate McLennan, Melanie J. Rock, Emma Mattos, Ann M. Toohey

**Affiliations:** ^1^Department of Community Health Sciences, Cumming School of Medicine, University of Calgary, Calgary, AB, Canada; ^2^O’Brien Institute for Public Health, Cumming School of Medicine, University of Calgary, Calgary, AB, Canada; ^3^Calgary Seniors Resource Society, Calgary, AB, Canada; ^4^Brenda Strafford Centre on Aging, Cumming School of Medicine, University of Calgary, Calgary, AB, Canada

**Keywords:** social welfare, pets, older adults, aging-in-place, health promotion, age-friendly communities

## Abstract

At the convergence of population aging and pet-ownership, community stakeholders are well-positioned to support older adults’ relationships with companion animals through age-related transitions in health and living arrangements. In this study’s setting, a volunteer-based pet care assistance program launched in 2017 to provide practical assistance with pet care for socially disadvantaged, community-dwelling older adults. This case study explored the impacts and feasibility of this and similar programs via (i) an Internet-based environmental scan to compare similar programs and (ii) qualitative interviews with a sampling of diverse community stakeholders (*n* = 9). A small number of comparable international programs (*n* = 16) were found. Among these, programs were delivered using a range of funding models; fewer than half involved collaborations across human social services and animal welfare sectors; and none addressed all dimensions of support offered by our local program. Analysis of qualitative interviews highlighted five major themes confirming the value of the volunteer-based approach and the importance of cross-sectoral collaborations in addressing older adults’ under-recognized pet care-related needs. Taken together, the findings confirmed the effectiveness of our local program model. Collaborative, cross-sectoral programs that target both human and companion animal well-being hold promise to reduce barriers to pet ownership that many disadvantaged older adults face. This unique approach leverages the health-promoting potential of human-animal relationships in ways that enhance quality of life for individuals, animal welfare, and age-friendliness of communities.

## Introduction

At the convergence of population aging and pet-ownership, community stakeholders are well-positioned to support older adults’ relationships with companion animals through age-related transitions in health and living arrangements. However, relatively little scholarly work has been written about health promoting opportunities that can be addressed by community-based programs that target human-animal relationships for older adults [exceptions include Rauktis et al. (2017); Toohey et al. (2017), and Cryer et al. (2021)]. Such programs are positioned to have positive impacts that also cross species lines, as they aim to simultaneously support both human health and well-being and animal welfare. Our case study fills this gap in knowledge in two ways. First, it offers insights derived from an environmental scan investigating how volunteer-based pet care assistance programs are delivered and assessing their impacts. Second, it presents a longitudinal assessment of an innovative program that was piloted in 2017 by a local charitable organization. This program was designed to align with a recognized community need and was built on a solid base of evidence (Toohey et al., 2017). In following the evolution of this program, qualitative interviews with key stakeholders were conducted to garner helpful insights after 4 years of program delivery. Moreover, this study contributes to a growing recognition of human-animal relationships as an often-overlooked dimension of “age-friendly” communities.

Core values of age-friendliness are reflected in efforts to promote independence and social inclusion of older adults by supporting aging-in-place (Menec et al., 2011; Steels, 2015). Ideally, aging-in-place policies recognize the functional, symbolic, and emotional attachments that older adults have to their homes and neighborhoods. Such policy efforts aim to enable older adults to lead meaningful and healthy lives while remaining in their communities for as long as possible (Menec et al., 2011). Yet few initiatives to promote age-friendly communities or support aging-in-place recognize (i) people’s desire to continue to have pets later in life, as is confirmed in the literature [see for example McNicholas (2014) and Bibbo et al. (2019)], and (ii) the health-promoting potential of human-animal relationships from a wider public health perspective [see for example Toohey et al. (2013); Rauktis et al. (2017), Toohey et al. (2017, 2018), and Toohey and Rock (2019)]. Our failure to consider the individual and systemic barriers that older adults may face when it comes to caring for their pets later in life also risks disrupting the health promoting potential of pet keeping (Gee and Mueller, 2019; Obradović et al., 2020). Given that on average, one-third of older adults in Canada and other countries report having companion animals (Toohey et al., 2017, 2018), the implications of both the potential collective benefits and the prospective harms of this oversight are notable.

Research findings offer valuable insights into the benefits of human-animal relationships for older adults. For instance, a recent scoping review of scientific and gray literature on companion animals and the health of community-dwelling older adults found that nearly half of the reviewed publications reported positive psychological outcomes such as increased feelings of happiness, self-efficacy, and relaxation, and social benefits such as decreased loneliness and isolation (Obradović et al., 2020). Companion animals can also encourage physical activity and facilitate interaction with the broader community through activities such as dog walking (Toohey et al., 2013; Curl et al., 2020) and socializing around shared interest in people’s cats (Mahalski et al., 1988). Research also suggests that in the home, older adults who spend time in the company of their pets may have improved mental health outcomes (Bennett et al., 2015), although the salience of such domestic interactions with pets for health and quality of life is often ignored by researchers (Ryan and Ziebland, 2015).

Relationships with companion animals can also pose significant challenges, especially for older adults experiencing socio-economic disadvantages, health challenges, and social isolation (Toohey et al., 2017; Toohey and Rock, 2019). Older adults living on fixed incomes, such as old-age pensions, may be forced to choose between fulfilling their own needs and those of their pet. Indeed, research has shown that older adults may negotiate challenges and even go to great lengths to maintain their relationship with a companion animal (Rauktis et al., 2017; Toohey and Rock, 2019; Applebaum et al., 2021a). For example, pet-prohibitive rental housing policies may force older adults into unstable housing (Ormerod, 2012; Toohey et al., 2017; Toohey and Rock, 2019; Matsuoka et al., 2020), or see them staying in unsafe situations (Toohey and Rock, 2019). Veterinary care may be financially inaccessible for older adults living in disadvantaged circumstances, yet withholding medical care is considered to be neglect and may lead to seizure or relinquishment of the animal (Alberta Veterinary Medical Association, 2019; Rock et al., 2020). Taken together, these different barriers point to a need for systems-level supports, including more pet-friendly affordable housing and both financial and material support for accessing veterinary care. Investments in these types of programs could leverage the prospective health benefits of animal companionship for older adults.

As a means of understanding mechanisms by which human-animal relationships may contribute to the health and well-being of older adults, Putney’s relational ecology framework is helpful. This framework is built upon the theoretical premises that human-animal relationships may mirror ecological interdependencies, enabling older adults to adapt to aging through the evolution of self-identity while influencing older adults’ definitions of self; contributing to developing and maintaining feelings of stability, security, and safety; and providing continuity through transitions that occur later in life (Putney, 2013). Qualitative research by Toohey et al. (2017) extended the relational ecology framework by demonstrating how older adults in socio-economically disadvantaged circumstances may face inordinate contextual barriers that shape their relationships with companion animals. These barriers align with different socio-ecological domains of intervention, including interpersonal, community, and policy-level influences (Richard et al., 2011). Furthermore, the increased likelihood of encountering such barriers can be linked to a relational understanding of individual autonomy and other underlying ethical concepts (Baylis et al., 2008). Informed by these theoretical underpinnings, the intent of this study is to offer practical insights into community programs that simultaneously address human and companion animal health and well-being and contribute to social justice by offering assistance with pet care.

Our particular focus is upon lower income, socially isolated older adults, who are more likely to face both inter-personal and systemic barriers that risk disrupting the health-promoting potential of pets and that also place animal welfare at risk. We also note, however, that over 37% of Canadians 65 years and older have a disability or chronic illness (Morris et al., 2018). While older adults may not self-identify as disabled (Kelley-Moore et al., 2006), older pet-owners who are also members of underserved populations will inevitably include those with disabilities and chronic illnesses [e.g., Toohey and Rock (2019)].

## Materials and Methodology

This study represents a deep exploration of a single case within a multiple-case study (Yin, 2009) designed to explore the health promotion implications of aging-in-place with companion animals (see Figure 1). Specifically, we draw upon knowledge generated in previous work to focus upon a volunteer-based pet care assistance program for lower-income and socially isolated older adults who are aging-in-place in an urban setting in Calgary, Alberta, Canada. Because of the absence of published literature on this type of specialized and relatively rare community-based program (Toohey et al., 2017; Obradović et al., 2020; Cryer et al., 2021), the first component involved an environmental scan for such programs, both to assess the prevalence and format of pet assistance programs for older adults. Next, we garnered the perspectives of community agencies involved in cross-sectoral collaborations in Calgary whose staff and volunteers deal directly with supporting older adults’ relationships with their companion animals. This important source of knowledge is underrepresented within the study of companion animals and aging. Ethical clearance for this study was granted by the Conjoint Health Research Ethics Board at the University of Calgary (REB14-1347).

**FIGURE 1:** Multiple, embedded case study design and scholarly outputs. Note that this study reports on findings from Unit of Analysis #3, while other scholarly outputs are listed within the figure.

### Calgary’s “Pet Assist” Program

Calgary has attained an international reputation as a model “pet-friendly” city [e.g., Rock (2013), Rock et al. (2014), and Economy and Infrastructure Committee (2016)], although its limitations, particularly the shortage of pet-friendly rental housing, have also been recognized (Toohey and Krahn, 2018; Graham and Rock, 2019). As an innovative program that operates outside of government, the Pet Assist program aims to fill some of the recognized gaps in supports for pets. The program is delivered by the Calgary Seniors’ Resource Society (CSRS), a registered charity that combines social work and professional services with volunteer programming and community engagement to support aging-in-place for low income, socially-isolated adults 65 years and older (Calgary Seniors’ Resource Society, 2021). Leading up to introducing this innovative program, CSRS staff and leadership had recognized the connection between quality of life and companion animals experienced by many of their clients, but were often unable to intervene appropriately when pet care challenges arose (Toohey et al., 2017).

Pet Assist was launched in 2017 and the urgency for this type of program is growing, given recent changes in policies of reporting medical neglect (Alberta Veterinary Medical Association, 2019) that may often reflect financial barriers to veterinary care rather than negligence (Rock et al., 2020). Pet Assist is delivered at no cost to clients. In addition to volunteer-delivered care, the program itself was built upon a foundation of fundamental cross-sectoral partnerships that were initiated with local animal shelters and rescue organizations, veterinarians, and the pet industry. The pet care support services offered span different species of companion animals (e.g., dogs, cats, birds, and others), and include practical assistance with dog walking, litter box or cage cleaning, and minor grooming; obtaining pet food and supplies; transportation to veterinary clinics; temporary boarding; and, on a case-by-case basis, subsidizing costs of veterinary care. This program also provides an opportunity for older adults to form relationships with volunteers through shared love of animals. While implemented by a social services agency, the program works at the interface of human and animal well-being by facilitating multi-sectoral collaborations that cross species lines.

### Environmental Scan for Comparable Pet-Assistance Programs

#### Case Selection

Programs similar to Pet Assist were defined as volunteer-based programs delivered at no cost to clients that support community-dwelling older adults with pet-related care needs. Prior to beginning the environmental scan, detailed inclusion and exclusion criteria were identified by the research team with reference to the evidence-based qualities of the Pet Assist intervention model. The inclusion criteria for programs found in the search were: (i) located in English-speaking countries, (ii) offered practical assistance for pet care at no cost to program users, and (iii) the target demographic was older adults living in the community. Programs identified during this search were excluded if: (i) they did not offer a broad scope of practical assistance (i.e., provided only one of the following: pet boarding, veterinary care funding and/or services including grants for animals that are critically ill, injured, or have cancer or pet food, or else the website did not identify what types of practical assistance are offered); (ii) they did not target the population of community-dwelling older adults with companion animals (i.e., programs for assistance and/or therapy pets only, a fee-for-service funding model with no subsidies, programs for senior and/or elderly pets, programs for pet owners experiencing homelessness, programs for pets of residents of long-term care facilities, programs for pet adoption, or programs for “community dogs” who did not have individual owners); and (iii) the program website did not mention supporting the wellbeing of the older adult in addition to supporting the welfare of the animal.

#### Search Strategy

A searching mode (Choo, 2001) was used by actively entering the Internet-based environment to collect data based on the inclusion and exclusion criteria detailed above. A research librarian was consulted for guidance with searching web-based data using rigorous methods. The environmental scan was conducted by KM over the course of 4 days during May 2021.

The environmental scan began with hand-searching reference lists of research publications known to the researchers that studied or mentioned specific pet support programs for older adults. The next phase of searching was open and iterative and conducted using the Google search engine. Initially, search terms were broad (e.g., *“pet care support seniors”*) then they gradually became more focused by including terms for regions of interest (e.g., *“pet support programs Melbourne Australia”*), and including different terminology for older adults (e.g., *“elderly, senior, aged”*). The websites that resulted from these search terms were thoroughly searched for information on the defined inclusion criteria.

#### Data Extraction

KM led the initial data extraction step. Data describing the criteria of interest were extracted by reviewing online program newsletters, financial reports, media, and testimonials from program users, and by following other recommended links that were provided on the program websites. In the cases of websites where detailed information could not be found, searches for the program name were done under the Google News function. In some cases, once programs were identified, searching them by name uncovered more websites of interest. As a final approach to identifying relevant programs, Op-Ed articles and blog posts about pets and seniors were searched. KT consulted with AT when uncertainties arose around either inclusion of appropriate data sources or alignment with data extraction criteria.

#### Data Analysis

To make meaningful comparisons, dimensions of programming that were considered included: the types of practical supports offered to companion animals and people; the number of older adult clients beings served; funding structures; volunteer base; and collaborations between human social agencies and animal welfare organizations. Data describing these different dimensions were entered into a tabular matrix (Miles and Huberman, 1994) that was developed by KM and refined collaboratively with AT. KM led the meaningful synthesis of data across programs within the criteria of interest described above. KM’s analytic decisions were confirmed or refined through deliberations with AT. This primary data is available by request to the authors.

### Qualitative Interviews With Local Stakeholders

#### Research Setting

Calgary has previously been recognized as a “pet-friendly” city based in part on municipal policies on responsible pet-ownership (Rock, 2013) and this city has been the setting of several components of the larger case study exploring the health-promoting potential of older adults’ relationships with companion animals. Calgary also launched an age-friendly municipal strategy in 2015, which emphasizes social inclusivity of older adults and is attentive to those living in vulnerable circumstances, including lower household income and social isolation (City of Calgary, 2015). In April 2019, the Alberta Veterinary Medical Association (ABVMA) instituted a policy for mandatory veterinary clinic reporting of animal abuse and neglect that local veterinarians must comply with (Alberta Veterinary Medical Association, 2019). Although instituted in the interest of animal welfare, this policy in combination with high veterinary costs may subject lower-income pet owners to reports of medical neglect and, in extreme cases, permanent seizure of the pet if the owner is unable to afford necessary veterinary medical care for their companion animal.

#### Sampling Strategy and Description

Our sampling strategy for interview participants was purposive in that we sought perspectives that could reflect on the need, feasibility, and impact of the Pet Assist program via relevant experiences. Calgary Seniors staff, volunteers, and community partners who work directly with the Pet Assist program were eligible to participate. Potential participants were recruited by a staff member of Calgary Seniors’ Resource Society (EM) based upon their familiarity and involvement with the Pet Assist program. Prospective participants recruited in this way were contacted via an email communication from this staff member and were invited to contact academic members of our research team (AT and KM) if they were interested in participating in the study. Additionally, potential interviewees with parallel interests in human-animal relationships but not necessarily working directly with the Pet Assist program were identified within the professional networks of MR and AT and were contacted via email by AT regarding the study and inviting their participation. Our final sample consisted of two program volunteers, one social worker employed by Calgary Seniors, and six individuals representing two local animal welfare organizations (Table 1).

**TABLE 1:** Description of participants interviewed as part of a case study exploring the need, impact, and feasibility of Pet Assist.

Description of represented organization	ID/Description
Social support agency (not-for-profit organization)	P1/volunteer
	P7/employee, social worker
	P9/volunteer
Animal welfare agency (shelter and other services)	P2/employee, executive director
	P3/employee, operations and protection
	P4/employee, animal operations
	P5/employee, animal operations
	P6/employee, support services
Animal welfare foundation (funder)	P8/volunteer

We obtained informed consent from each participant. Three individual interviews and one group interview were conducted over both Zoom and one individual interview was conducted by telephone. Each interview lasted 30–60 min. The interviews were semi-structured, with discussions supported by interview guides developed by our research team. Interview guides were designed based on previous knowledge of the Pet Assist intervention as well as evidence on the benefits and challenges of aging-in-place with pets, and each was tailored to each participant’s role and/or involvement with the Pet Assist program.

AT and KM conducted all interviews between June and July 2021. All interviews had two researchers and one participant present except the group interview conducted with Participants 2–6, who represented different operating arms within a major local animal welfare organization. The interview with Participant eight was conducted by telephone and was not audio-recorded at the participant’s request. Extensive field notes were taken, then reviewed and approved by the participant. All other interviews were conducted virtually using a secure Zoom connection and were recorded for transcription with participants’ permission. Members of the research team wrote field notes during interviews and research memos immediately after each interview (KM and AT) and during the transcribing process (KM).

#### Data Analysis

The interview recordings were initially transcribed using digital software offered by Zoom^®^, and each automated transcript was reviewed and corrected by KM in the style of verbatim transcription. During this process, KM also wrote research memos to capture initial impressions, questions, and comparisons within and between each interview. Data were reviewed multiple times by KM as she progressed through an iterative and reflexive process of semi-inductive thematic analysis (Braun and Clarke, 2006, 2020). The analytic approach was semi-inductive as interview questions had been organized around broad interests in the perceived need for and impact of pet care assistance programs for older adults, as well as issues concerning the feasibility of delivering these unique but complex offerings. Through an immersion and crystallization process (Borkan, 1999), KM expanded understandings of manifest themes identified during initial coding, leading to an understanding of latent themes. KM continued to refine themes based on iterative and evolving insights surrounding the data and through discussions with AT, based on both impressions of the interviews conducted and understandings garnered from previous components of the case study of the health-promotion potential of aging-in-place with companion animals. The other authors (EM and MR) reviewed the proposed analysis from their own understandings of the program. EM contributed practical expertise in navigating the landscape of social support programming for disadvantaged older adults in Calgary, while MR offered scholarly expertise in the underlying theories that inform health promotion via policy-level interventions involving companion animals (Rock, 2013, 2017).

## Results

### Environmental Scan

In total, 59 international programs were found and 16 of those met the inclusion criteria defined in the methods section Case Selection. Thirty-one programs were excluded because they did not offer a similar scope of practical assistance. Within those programs, ten offered one-time grants for animals with cancer or other critical injuries and illnesses. The remaining 12 programs were excluded because they did not target the same demographic of community-dwelling older adults living with companion animals. Of the included programs, one was located in Canada with services for dog care available in nine provinces, three programs were located in the United Kingdom with services available in England, four programs were delivered in the United States with services available in eight states, and eight programs were found in Australia with services available in five states. Every program was aimed at supporting community-dwelling older adults with a companion animal.

Comparisons across the different programs reviewed are summarized in Table 2. All programs targeted older adults and half of the programs (USA-1, 2; UK-1; AUS-1, 4, 5, 7, 8) had minimum age requirements ranging from 55 to 65 years old, however many programs also accepted younger people with disabilities or terminal illness. Every program offered practical assistance with support such as dog walking, litter box cleaning, grooming, and transport for veterinary care, all provided by volunteers. Several programs (USA-2, 4; AUS-5) offered limited financial support for veterinary care and pet supplies on a case-by-case basis. One program in the United States provided practical assistance and lifetime sponsorships for 50 pets whose owners met income cut-off eligibility requirements (USA-1). Nearly half of the programs (UK-2, USA-3, AUS-1, 2, 4, 7, 8) explicitly mentioned the importance of fostering social connection and inclusion of older adults in their communities, and most programs made a general comment about the importance of the human-animal bond and research that has linked pet ownership with health benefits. One program in the United Kingdom (UK-2) and six programs in Australia (AUS-2, 3, 4, 6, 7, 8) provided information on the training that volunteers receive. The most rigorous training included dog behavior, safe relationship boundaries between older adults and volunteers, suicide awareness, and communication skills (AUS-6).

**TABLE 2:** Comparison between dimensions of the Pet Assist model and dimensions of comparable programs found in the environmental scan.

Dimensions of the Pet Assist Model	Pet Assist	CAN-1	UK-1	UK-2	UK-3	USA-1	USA-2	USA-3	USA-4	AUS-1	AUS-2	AUS-3	AUS-4	AUS-5	AUS-6	AUS-7	AUS-8
Dog-walking	X	X	X	X	X	X	X	X	X	X	X	X	X	X	X	X	X
Litter box maintenance	X		X	X		X	X	X	X	X	X	X	X	X			X
Obtaining pet supplies	X	X	X			X	X	X	X	X	X		X				
Minor grooming	X	X			X	X	X	X		X	X	X	X	X	X		X
Animal transport	X	X		X	X	X	X	X		X	X	X	X	X	X		X
Temporary boarding	X	X	X	X	X									X			
Relationship building with volunteers	X			X				X		X	X		X			X	X
Collaboration with animal welfare	X			X		X	X		X				X	X	X		
Not income-regulated	X	X	X	X			X	X	X	X	X			X			X
Age-based eligibility	X			X	X	X	X			X				X	X	X	
Accepts multiple pet species	X		X	X		X	X	X	X	X	X	X	X	X			

*CAN-1, Elder Dog Canada; UK-1, Cinnamon Trust; UK-2, Keep Your Pet-Age UK; UK-3, The Light of the World Trust; USA-1, The Kado Pet Foundation; USA-2, PAWS/LA; USA-3, Pet Pals-Sunnyside Community Services; USA-4, Pets and Elders Together-Search and Care; AUS-1, LinkPETS-Link Health & Community; AUS-2, Pets for Life-Caloundra Community Centre; AUS-3, Pet Companion Program-Bridges Connecting Communities; AUS-4, Pets of Older Persons (POOPs); AUS-5, Community Aged Care Program-Royal Society for the Prevention of Cruelty to Animals New South Wales; AUS-6, The Companion Animal Project-City of Charles Sturt; AUS-7, PetMates-South Port Day Links; AUS-8, Companion Animal Volunteer Support-Balwyn Evergreen Centre.*

A notable finding from the environmental scan was that none of the comparable programs provided all the dimensions of support offered by Pet Assist (Table 2). Additionally, Pet Assist is the only program of its kind in Canada that offers supports to socio-economically disadvantaged older adults with pets of all types (i.e., a non-species-specific program, as opposed to dog- or cat-specific supports).

#### Funding Models

All programs in Canada, the United States, and the United Kingdom were funded by charitable donations from individuals and corporations. One program in the United States (USA-3) was funded by a pet-related foundation started by a social worker, and another program received a small amount of funding from a municipal government’s department of aging (USA-4). One program in the United Kingdom (UK-2) was funded by a local charity for supporting seniors, which in turn was funded by municipal grants, charitable grants, and donations from the public. Six of the eight programs in Australia received both state and federal government funding and older adults can apply for these programs through a government-run online portal for an array of services for older people (AUS-1, 2, 3, 6, 7, 8). One of the programs in Australia (AUS-2) has been funded by a family foundation since 2017 and four of the programs accept donations from the public and corporate sponsors (AUS-2, 3, 4, 7). Pet Assist’s funding model is the most similar to USA-3, which received funding from donations and limited funding from a pet-related family foundation (USA-3; SCS, 2018).

#### Cross-Sectoral Involvement

All programs in the environmental scan prioritized supporting older adults by supporting their relationships with pets; however, the programs differed in terms of the level of involvement between human social service and animal welfare agencies. Half of the programs had partnerships with veterinary clinics or veterinary nursing students (Can, USA-2, UK-1, 2, AUS-2, 4, 5, 6). One program in the United Kingdom (UK-1) employed an animal welfare consultant and another (UK-2) was run in collaboration with a local animal welfare agency. In Australia, one program (Aus-2) worked closely with an animal rescue organization and a university-anthrozoology research group. Another Australian program (AUS-5) was funded and delivered by an animal welfare organization.

In Australia, the Royal Society for the Prevention of Cruelty Against Animals (RSPCA) commissioned a toolkit on funding and implementing companion animal support programs (Alfonsi, 2016). This toolkit was evidence-based and developed with involvement of numerous stakeholders. The toolkit also referenced and discussed several programs identified in this environmental scan, including every Australian program and one large organization in the United States that provides companion animal support services through 13 affiliated programs across several states (USA-2).

For comparison, Pet Assist combines professional services from social workers employed by Calgary Seniors while partnering with the three other social services agencies. In addition to these supports from social services, Pet Assist collaborates with a local animal welfare agency to make use of the emergency boarding programs they offer, and they have received donations from a corporation in the animal care industry. Additionally, Calgary Seniors connects older adults using the Pet Assist program to a local lower-cost veterinary clinic.

#### Reported Impact

Some programs in the environmental scan reported quantitative metrics describing impact, such as the number of people and pets supported through the program, although these are difficult to compare due to inconsistent measures. For instance, the largest program in the United States served older adults with companion animals in 13 states (USA-2). The largest program in the United Kingdom reported serving 150,000 people and 157,977 companion animals per year (UK-1). The largest program in Australia reported serving 260 older adults and 300 companion animals since the program began (AUS-4). For comparison, Pet Assist served over 90 older adults with companion animals in 2019 and continues to grow.

Programs in the environmental scan also reported qualitative metrics for impact, such as testimonials from older adults published on program websites or in the media. One older adult receiving a lifetime sponsorship for their pet from a program in the United States reported that, “thanks to (the program), my kitties are safe and I don’t have to stress about how they are going to get fed or when they need to go to the vet…Funds are extra tight and I am no longer able to afford to take care of their financial needs” (The Kado Pet Foundation, 2021). An older adult using a different program in the United States reported that, “thanks to (the program) I am able to have and take care of Riley, who in turn really takes care of me” (PAWS/LA, 2021). A program in the United Kingdom published case studies, such as the story of an older adult who “…had been frail for some time. (Program) volunteers visited daily to take (the dogs) for their walks so they could remain with their mum who loved and needed them so much” (The Cinnamon Trust, 2021). This program also committed to rehoming the pets following this woman’s passing. The Pet Assist program also regularly includes testimonials from older clients in its publicity materials, including reports to donors, underscoring the impact of its volunteer pet care support on clients’ quality of life.

### Qualitative Interviews

In total, two program volunteers, one social worker, and six individuals representing two different animal welfare organizations were interviewed. Our interviews were designed to explore participants’ perspectives on the need, impact, and feasibility of the Pet Assist intervention. Our reflexive thematic analysis (Braun and Clarke, 2020) of the qualitative interview data led us to identify five major, recurring themes.

#### Theme 1: Just One More Thing We Do to Seniors

The first recurring theme recognized that the disadvantaged older adults receiving support from Pet Assist experience numerous structural inequities and are subject to endemic ageism [i.e., discrimination rooted in paternalistic prejudice and perpetuated by both positive and negative stereotyping of older adults (Cary et al., 2017)]. At a systemic level, participants recognized that rules and regulations implicit to eligibility for social assistance and affordable housing policies posed barriers to maintaining relationships with pets. Older adults depending on these programs and supports are also likely to experience adversity related to poor health and chronic illness that impeded their ability to care for their pet. As the social worker in our sample noted:

…if they do ask somebody for help, the automatic comment is—a lot of them will have children that are busy, they’re raising their families or whatnot, can’t come, and so the senior’s still isolated—and then it’s “you shouldn’t have (the pet),” right? (P7)

This perspective reinforces an implicit expectation that relationships with pets are dispensable for older adults, when challenges arise or circumstances change. And yet, a program volunteer also reflected that “it was a real eye opener to see someone that’s just living on, you know, government pension” (P9). This volunteer had never encountered the impoverished conditions like those of the older adult couple who she was supporting via dog-walking assistance. She felt that the experience had given her a much greater understanding of and empathy for the struggles her clients experienced on a daily basis. Linked to these insights was her recognition that being forced to part with their dog would be both devastating and unjust, given that the cherished pet—who also facilitated regular visits from the volunteer—was one of the few sources of joy in their lives. A similar sentiment was held by another program volunteer, who expressed that being forced to part with pets is “just one more thing we do to seniors that is improper” (P1). Notably, however, volunteers also felt that the Pet Assist program’s ethos reflected a high level of respect for the voice and choice of the older adults they were supporting. As one volunteer noted:

There’s a way to talk to them to get a good sense of where their needs might be without making them feel embarrassed or less than … (you) try the best you can to understand the perspective and you can work on that with simple conversations over tea (P1).

#### Theme 2: Intertwined Lives, Intertwined Quality of Life

The second theme from our analysis highlighted the extent to which both the lives and quality of life of older adults and their companion animals are intricately intertwined, and therefore both parties are impacted by the marginalization of disadvantaged older adults. Most participants recognized that the human-animal bond is highly valued by older adults and that without supports, they may sacrifice their own needs and health to maintain a relationship with their pet. For instance, based on her years of clinical experience, the social worker shared:

…many of the seniors, you do find that they will often not be seeking medical care because they don’t have assistance for the pets. So they don’t want to leave the pet behind or don’t have anyone to look after them, and they get stuck, right? … you have the ones that are going without their own food or their own medication, trying to keep up with looking after the (pet)… either because of money or because they don’t have the support to look after the pet (P7).

Participants also felt that older adults’ access to veterinary care is a significant consideration for maintaining a relationship with an animal and with the animal’s welfare. As one animal welfare employee mentioned, “The cost of vet care is also a concern. It is prohibitively expensive in Alberta …” (P4). In addition to cost, participants also noted both transportation as a common challenge and, along a more troubling vein, anxiety that older clients experienced around the prospect of facing discrimination related to socio-economic status:

There’s a reluctance to acknowledge things that are going wrong with the pets and they just don’t see it. It’s daunting for them to think about getting in the car—if they have a car, if they’re able—and going to a vet clinic, being looked at that way. I know my first [client] was sensitive to being seen as low income… (P1)

These barriers were viewed by some participants as putting older adults at risk of perpetuating varying degrees of medical neglect, with unintended consequences for the welfare of their pets. Participants representing a major local animal welfare organization suggested that medical neglect “…was by far the largest increase in reason for intake, based on the number of animals admitted to the shelter…” (P2).

The Pet Assist program, however, was also recognized as an importance means of intervening before issues of health and quality of life overwhelmed. The social worker spoke of the importance of the whole program:

…they already have their own things going on but worrying about their pet and medical conditions or whatnot, so when they actually get into the program, and someone comes and assists to walk and assists to feed their pet, the stress level goes so far down. And you’re talking people in crisis, so it’s just another added layer of what a senior has to deal with when there’s already so many issues going on (P7).

An animal services representative also shared that “one of the biggest barriers that a lot of seniors will face to getting that appropriate care (for their pet) is quite simply that: transportation,” also noting that “…it’s all connected, right? So we want to see the people taken care of too. They can’t take care of the animals unless we’re taking care of the people” (P3).

#### Theme 3: Continuity in the Face of Adversity

A third recurring theme captured the view that older adult’s relationships with their companion animals offer a semblance of continuity in the face of adverse events such as loss of employment, loss of health, and loss of relationships. Participants consistently recognized that having a pet to care for enabled older adults to sustain a sense of purpose and establish a routine, even as other parts of their lives devolved in various ways:

It’s really (about) allowing that dog to remain’ cause she has nothing else left … you know, the inability to go out and even walk normally let alone partake in activities or be social, get out, do all of that. All of that is gone for that for that couple, so what remains really, over and above each other and television, is the pet. And they’ve had that pet for 8 years, it’s not like they just got it last week…” (P1)

Several participants also commented on ways that pets helped to ameliorate experiences and impacts of social isolation in relation to a sense of continuity that might otherwise be supported by human relationships:

For most of them it’s amazing that they’ll tell you that’s their reason for getting up in the day, that’s where they get their exercise, that helps them to keep, you know, moving and doing different things… and then isolation is, I mean, that’s the biggest reason, right? They don’t have that social network with those supports (P7).

As an important dimension of receiving pet care support, relationships that program clients established with volunteers were also understood to contribute to experiences of continuity, including the prospect of clients losing their cherished pet:

…I know for a fact she would be calling me up, wanting to talk. I mean she calls me just to see how my day’s going … so when the day comes I would ask (the program) if I could continue to be involved with her … I think it’s important for that continuity of care to sit and reminisce, because now you have that shared experience with your senior where you’ve also experienced a relationship with that dog, so I think it could comfort in sharing that grief (P1).

Both volunteers interviewed expressed a desire to maintain their relationships with the older adults they were currently assisting with pet care, even beyond the currency of their pet-related needs.

#### Theme 4: A Critical Lifeline Keeping People and Pets Together

A fourth theme reflects the perspective that the support offered by the Pet Assist program is a critical lifeline for keeping people and pets together. Pet Assist offers a wide range of pet-specific supports, but that also include social connection with volunteers, and transport and support for veterinary care. There was a prevailing view that older adults work very hard to care for their companion animals and oftentimes minimal support is needed to keep people and pets together. However, needs can change acutely and suddenly in older adults’ lives, whether temporarily or permanently. Participants highlighted the importance of the comprehensive dimensions of support that are offered through Pet Assist. As one volunteer reflected, “She thanks me almost every time I’m there for, you know, making it possible for them to keep their dog” (P9). The other volunteer shared that “the problem is literally with being able to give that dog what is needed, and if we weren’t there to walk that dog it would have to be taken away” (P1). The social worker also noted that in her experience:

There are so many seniors out there that could continue looking after their pets. They’re more than willing, they’re able … and a lot of times it’s temporary situations, they’ve had some type of health issue, it’s just a temporary, but not having that support means all of a sudden they’re gonna lose their pet” (P7).

Finally, without the pet care supports provided by the Pet Assist program, it was felt that more older adults would be forced to relinquish their pet or make undue sacrifices:

… you can tell that they really do care for these pets and they’re trying their absolute best to get them everything that they need, but they have these just natural barriers as a result of, you know, growing older that they’ll face and encounter. So we do see that in the admissions department relatively often (P3).

#### Theme 5: Building Connections That Cross Species Lines

The final theme identified across the interviews illustrated the invaluable opportunities that result when connections that cross species lines can be made, as a crucial means of addressing challenges that involve both human and companion animal considerations. The participating social worker noted “I think there’s a lot of people out there that would be more than happy to help walk a dog or stop by and, you know, change the kitty litter and stuff if they knew” (P7), while the volunteers also felt that many people would be interested in volunteering for a program like Pet Assist if they knew of the “need unspoken” (P1) that exists in the community. Along similar lines, an animal welfare representative also reflected that older adults with more expansive social networks than the Pet Assist clients might receive supports that were “…kind of, you know, organic, where neighbors or friends and family kind of (assist)” (P3). Pet Assist was unequivocally recognized for making opportunities for relationships with companion animals more equitable for those older adults who don’t have access to these types of social supports in their lives, while also being rewarding for volunteers.

Furthermore, the opportunity to assist with pet care was viewed as having reciprocal benefits for those providing the help: “I love to walk and I love pets so it was a good combination…it’s a good relationship and, you know, it’s good for me and for them” (P9). Similarly, an animal welfare representative noted that “I think that shared responsibility around animals is wonderful and I think a lot of people feel very lucky when they get to participate in it” (P5). This view was also expressed by another animal welfare representative, in reflecting on volunteers involved in the emergency temporary foster programs that are sometimes accessed by Pet Assist:

Particularly for those animals in the Pet Safekeeping or Emergency Boarding programs, when they are owned animals with people who are facing some pretty significant hardship in their life, they feel so lucky that they get to take in that animal and care for them until their owner is ready to take them back (P5).

There was a concern voiced among several of the participants that many professionals working in animal welfare and social services are unaware of programs like Pet Assist. It was suggested that this lack of awareness contributes to the pervasive, systems-level view that older adults should relinquish their pets to a shelter or an acquaintance should they experience difficulty caring for them for any reason. As suggested by one of the animal welfare representatives:

(We) might look at the intake diversion portion of [Pet Assist] because if in fact there was a service out there that could provide transportation for the animal to a private veterinary clinic rather than seeking [our lower cost veterinary services], that would be super helpful and that would allow us to keep animals from being potentially surrendered (P3).

The Pet Assist program’s innovative program design and effectiveness at fostering connections, via both cross-sectoral collaboration and opportunities for volunteers to assist with pet care, contributed to its success. Uniquely positioned to address human and companion animal needs simultaneously, Pet Assist was credited with enhancing the health and well-being of both older people and their pets.

## Discussion

This study aimed to understand the role that community stakeholders play in promoting the health and well-being of disadvantaged older adults by delivering volunteer-based pet care support programming. Our environmental scan confirmed that the need for this type of programming has been recognized in several countries world-wide. Furthermore, demand for pet care assistance programs inevitably exceeds the scarce program-based supports that are available, as captured within our interview data. Most comparable programs are delivered by charitable organizations, with Australia’s state-level funding support for programs that nurture human-animal relationships being unique and innovative. Positive impacts on both older adults’ quality of life and animal welfare, as described by case studies and testimonials, confirm the effectiveness of varied approaches to delivering pet care support. It is also relatively common, albeit not ubiquitous, for such programming to involve cross-sectoral collaborations between social services and animal welfare organizations. Even when compared with the other international programs we reviewed, our own local program stood out as particularly innovative, given the breadth of support delivered and the extensive foundation of both human social support and animal welfare expertise upon which the program is built.

Our qualitative interviews allowed us to gain in-depth insights into dimensions of the Pet Assist program that position it to be both effective and feasible. More specifically, Pet Assist was described by interview participants as being both novel and impactful for (i) integrating organizational values of inclusivity and social justice into a program offering that recognizes the valued, health-promoting roles pets often play in the lives of socially isolated older adults; (ii) establishing fundamental and reciprocal collaborations between human social services and animal welfare sectors as an effective and feasible means of providing vital support to the lower-income demographic of older adults, who often face intersecting forms of disadvantage like social isolation and chronic illness; and (iii) offering a compelling and unusual volunteer opportunity that merges interests in supporting older adults needing help with affinity for pets and concern for animal welfare. Moreover, Pet Assist contributes to the age-friendliness of our urban community by supporting independence and inclusion of socially disadvantaged older adults for whom aging-in-place can be a challenging prospect. Such older adults are regularly marginalized and expected to give up their pets in order to be eligible for supports like affordable housing (Ormerod, 2012; Toohey et al., 2017; Toohey and Krahn, 2018; Toohey and Rock, 2019). Pet Assist, however, acknowledges the importance of human-animal relationships in the lives of *all* older adults, including those who face social and financial disadvantages. Offering affordable assistance with pet care sustains these relationships for as long as it is safe to do so, and also connects socially isolated clients with compassionate human relationships and access to additional services and supports.

Confirming the need for pet care assistance programs, our thematic analysis illustrated the program’s ability to address real barriers and gaps in support that often disrupt older adults’ abilities to maintain valued relationships with companion animals. For instance, our analysis confirmed previous research findings that socially isolated, lower-income older adults face numerous systemic inequities that limit their ability to have companion animals (Rauktis et al., 2017; Toohey et al., 2017; Toohey and Rock, 2019; Matsuoka et al., 2020; Applebaum et al., 2021a,b). Our findings also demonstrated how the impact of these inequities introduce precarity into human-animal relationships later in life and thus put at risk the well-being of both people and pets. As circumstances shifted, human and animal needs were seen as becoming inextricably connected and requiring interventions that could address both simultaneously. The importance of addressing the needs of both people and their pets together has been observed in other studies as well (Rock and Degeling, 2015; Toohey et al., 2017; Toohey and Rock, 2019).

With the Pet Assist program targeting human-animal relationships, the volunteer-based pet care intervention was recognized as having far-reaching and intertwined impacts on older adults and their companion animals. Findings illuminated the potential of such interventions to benefit both human well-being and animal welfare. Our qualitative interviews underscored ways that supporting relationships with pets provided older adults with a means of navigating challenging life transitions, including coping with disability and chronic illness. Participants described how pet care assistance programs were able to protect animal companionship, maintain meaningful daily routines, and sustain deeply-felt responsibilities of having a pet, as has also been highlighted by others (McNicholas, 2014; Toohey et al., 2017; Bibbo et al., 2019; Toohey and Rock, 2019; Applebaum et al., 2021b). Pet Assist was viewed as being well-positioned to mitigate seizures or relinquishments of pets related to the condition of the animal, which was often at risk due to factors like costs of veterinary care or challenges with transportation to veterinary clinics, rather than negligence on the part of the older pet owner.

The feasibility of the volunteer-based model and cross-sectoral collaboration that takes place through Pet Assist program delivery was also confirmed by our interview participants. Feasibility was recognized both in terms of implementing a program that appealed—and was perceived as rewarding—to volunteers and for reciprocating the value of cross-sectoral partnerships for achieving the mandates of both human social service and animal welfare organizations. From a feasibility perspective, the environmental scan findings also offered valuable insights into new funding models, training approaches, and partnerships that could be replicated and tailored by both existing and future pet care assistance programs aimed at keeping older adults and their pets well—and together. An important, practical outcome of conducting this study was an unanticipated opportunity to strengthen the relationship between a major local animal welfare organization and the Pet Assist program. In conducting interviews with representatives of this organization, members of our research team recognized new opportunities where reciprocal benefits were likely and facilitated additional meetings between the two organizations. At the time of preparing this manuscript, both organizations’ abilities to achieve respective programming goals have been strengthened, and future collaborative plans are being actively developed.

Given the inordinate challenges that socially disadvantaged older adults face when it comes to having pets later in life, there is value considering the relational public health ethics framework for its relevance to matters of social justice (Baylis et al., 2008; Rock and Degeling, 2015; Toohey and Rock, 2019). Specifically, a relational ethics perspective posits that access to health-promoting opportunities will be inequitably distributed across the population, in relation to social position and access to both material and social resources. Recognizing the potential of human-animal relationships to support well-being as being both relational and subject to social disadvantage confirms the value of applying a relational socio-ecological understanding to the phenomenon. Systemic considerations that lead to the precarity of pet-ownership experienced by disadvantaged older adults who are aging-in-place with pets are gradually being recognized in relation to social justice [e.g., Rauktis et al. (2017), Toohey et al. (2017), Toohey and Krahn (2018), Toohey and Rock (2019), and Matsuoka et al. (2020)], yet merit continued study, particularly within efforts to create age-friendly and inclusive communities.

### Recommendations for Practice

The findings of this study have confirmed the need for pet care assistance programs for older adults and have offered evidence around impact and insights into the feasibility of such programs. Based on our findings, the value of creating meaningful and robust cross-sectoral collaborations between human social support and animal welfare organizations cannot be overstated. Animal welfare professionals can assist human-focused agencies in an array of ways, including involvement with producing and delivering volunteer-training modules as well as providing guidance and access to supports related to animal health and welfare. At the same time, as animal welfare organizations expand the scope and reach of their own programming into their local communities, organizations that have created infrastructures of support for older adults may be instrumental as partners or guides in addressing issues related to transportation, housing, mental health, and life transitions that older pet-owners may face. For instance, a report produced by the Vancouver Humane Society (2021) recommends integrating best practices from social services into animal welfare. Formal partnerships between social service and animal welfare organizations may also offer opportunities for financial efficiencies in addressing the needs of both people and pets.

The volunteers participating in this study reflected passionately on the personal rewards that they themselves experienced by helping older adults to care for their pets. The services they could provide addressed both their own connections with companion animals and their interests in serving older people in need of support. A similar experience was recognized by animal welfare professionals, who were attuned to the experiences of their own volunteers involved in emergency temporary fostering programs. The environmental scan uncovered numerous programs that offer grants for companion animals with critical illness, injury, and specific medical diagnoses such as cancer. The intrinsic motivations of volunteers might prospectively be further leveraged, and those with appropriate skills could help apply for appropriate grants with or on behalf of pet care assistance clients.

The costs of caring for companion animals may become increasingly challenging for lower income older adults living on fixed pensions. As one novel future approach, programs like Pet Assist could also support clients interested in fostering animals, rather than focusing exclusively on support for owned animals. Pet assistance for older adults who would like to help foster animals rather than take on full responsibility for a pet would offer flexibility and access to the benefits of the human-animal bond, and also create meaningful roles for those who are unable to afford to own their own pet. As another means of addressing the high costs of veterinary care, pet care assistance programs could explore negotiating discounted or group pet insurance for their clients, as a prospective solution to redressing inadvertent medical neglect of companion animals by reducing inordinate medical fees. Perhaps most importantly, however, the veterinary community’s involvement in ensuring that medical attention for pets can be made accessible and affordable for lower income pet owners is needed (Rock et al., 2020).

### Strengths and Limitations

There is a shortage of research on volunteer-based health promoting program that seek to protect human-animal relationships by providing assistance with pet care to older adults. This study is one of the few to explore such programs in the context of creating age-supportive communities, and therefore makes an important contribution. Strengths of this study include the collaborative involvement of the community partner that delivers the program (EM) in the study’s design to ensure that the findings have practical applicability for further evolving the program. This study also provides a deeper understanding of the lived experiences of socially isolated, lower income older adults with pets. Older pet owners’ socio-economic and social circumstances are rarely considered in research on human-animal relationships, and these relationships are rarely acknowledged as being relevant to organized efforts to promote the health of the aging population.

There are also important limitations of this study that must be considered. For instance, the environmental scanning methods may have been limited by variation in the quality and detail of information that was provided on the websites used to extract data. Data describing funding details, the number of program users, and eligibility requirements were not consistently available on each program’s website and were often garnered from secondary sources such as media coverage of the programs. The search was also limited to websites in English, and comparable programs from non-English-speaking countries may have been excluded.

The qualitative interviews included in this case study captured a breadth of perspectives but were conducted with a limited number of stakeholders. Additional perspectives of partnering organizations as well as both practitioners and volunteers involved with Pet Assist and other similar programs would offer additional valued insights. Furthermore, the voices of Pet Assist clientele were not included in this study due to issues concerning privacy and anonymity. Future studies could survey clients to better describe the challenges they have faced in relation to their pets and could confirm or expand upon the impacts to their lives that the participants in this study have observed.

Overall, our study’s findings point to the promise of pet care assistance programs as being both impactful and feasible. Such programs promote the health and well-being of socially disadvantaged older adults and their companion animals, contributing to social inclusion and social justice. Collaborative, cross-sectoral programs that target both human and companion animal well-being hold promise to redress barriers to pet-ownership that many disadvantaged older adults face. This unique approach leverages the health-promoting potential of human-animal relationships in ways that enhance quality of life for individuals, animal welfare, and age-friendliness of communities.

## Data Availability Statement

The datasets presented in this article are not readily available because qualitative interview data are available only to members of the research team as per the terms of participants’ informed consent; however, environmental scan data are available by request. Requests to access the datasets should be directed to AT, amtoohey@ucalgary.ca.

## Ethics Statement

The studies involving human participants were reviewed and approved by Conjoint Health Research Ethics Board (CHREB) at the University of Calgary (REB14-1347). The patients/participants provided their written informed consent to participate in this study.

## Author Contributions

KM conducted the environmental scan, supported qualitative interviews, transcribed recorded interviews, led the thematic analysis of environmental scan and interview data, and prepared an initial report on findings. AT developed the overarching methodology for the study, conducted qualitative interviews, provided iterative and substantive input into data analyses for both the environmental scan and interview data, and led preparation of this manuscript in its current format. MR provided direction on sampling and the scope of interviews and provided substantive input into early drafts of this manuscript. EM assisted with recruitment of participants and provided substantive input into early drafts of this manuscript. All authors contributed to the article and approved the submitted version.

## Conflict of Interest

The authors declare that the research was conducted in the absence of any commercial or financial relationships that could be construed as a potential conflict of interest.

## Publisher’s Note

All claims expressed in this article are solely those of the authors and do not necessarily represent those of their affiliated organizations, or those of the publisher, the editors and the reviewers. Any product that may be evaluated in this article, or claim that may be made by its manufacturer, is not guaranteed or endorsed by the publisher.
